The article "Research on the Development Path of Community Education Curriculum from Marx's Perspective Based on Big Data" was retracted in 2023. Reasons: unreliable results or conclusions; no approval from a third party; concerns about the data; concerns about the results or conclusions.

# Research on the Development Path of Community Education Curriculum from Marx's Perspective Based on Big Data

**DOI:** 10.1155/2022/9755391

**Published:** 2022-09-26

**Authors:** Zhila Sun

**Affiliations:** School of Marxism, Southwest Jiaotong University, Chengdu, 611756 Sichuan, China

## Abstract

Community education curriculum is the key link to achieve the goal of community education; it is an educational activity that uses the educational and cultural resources of the community and faces all residents in the community; promoting the innovation of community education curriculum is the new mission of the development of contemporary community education, in order to explore the development path of community education curriculum from Marx's perspective under big data and study its educational value and development path. By comparing the development paths of community education in different environments, this paper makes a comprehensive analysis and evaluation and analyzes the value of coupling degree. It can be seen that the use of big data technology has a positive impact on the development of new education models, the development of community education and platform management, and the learning motivation of residents. We should make breakthroughs and innovations on the basis of the traditional education model, realize the value concept of lifelong education, and follow Marx's socialist development concept; it can better promote the development of residents and communities in the community and provide more effective data value and data support for the development path of community education in the future.

## 1. Introduction

In the development path of socialism with Chinese characteristics, we should use the development direction of Marxism, Mao Zedong Thought, and Deng Xiaoping theory to achieve the development goal and strategic thought of building a well-off society in an all-round way. In the process of the development and progress of China's socialist society, the development and progress of the country need the joint efforts of the next generation and contemporary people, and it is also the most important node for the development and direction of learning education. Zhongbiao as an important part of adult education and community education in China implements the ideological quality of lifelong learning, and the idea of never too old to learn is a good quality [1]. The guidance and learning of community education courses are conducive to the cultivation of higher personal and social values and a sense of identity for our people. Caijinming summarized and analyzed the excellent education mode and teacher force applicable to the whole society through the education mode of Quanzhou Community University and built a community education path in line with local adult education according to the actual situation of each region [2]. According to Heqing and Yueheng, in the current era, the teachers of traditional community education gradually cannot keep up with the development speed of community education. The application of Internet big data technology can effectively deal with this situation. Based on big data technology, online education mode can be realized and more teaching forms can be adapted [3]. In the establishment of the community education model in the Yangtze River Delta, through the reasonable construction and framework of the education model, relying on regional advantages and the establishment of sharing mechanism to achieve multi-level and multi-type Education Division [4]. Rui implements the education concept of lifelong learning and realizes the education mode in line with national policies from the application and development of big data technology to the online world combined with the modern community education mode. With the help of digital resources, it is also conducive in improving the national economic and political level [5]. At the same time, the path method is applied to practice and compared with the traditional way of curriculum construction, so as to ensure that the construction and development of community education curriculum resources are more standardized, provide rich and high-quality curriculum resources for lifelong learning and learning city construction, and gradually improve the connotation of community education. According to Yanhong, with the serious aging situation in China, attention has been paid to the work of learning and reeducation for the elderly. With the development of digital technology, the addition and effect of community education have begun to take shape. In the future, it is necessary to solve the bottleneck and development path of community education by improving personal planning and striving for relevant national policies [6]. Jia has opened up a new path for the inheritance and development of China's intangible cultural heritage through the development mode and flexible application of community education [7]. According to Jing et al., community education is a policy-oriented cause. When the national policy is not perfect, there are still many defects in the development path of community education. In the future, the analysis and research direction of the development path need to be put forward [8]. This paper makes a comprehensive research and analysis on the development path of community education under the digital economic environment and the use of big data technology and perfects and develops the education mode in line with the concept of social development from the perspective of Marx; facing community residents, we should take the promotion of human development as the principle, so as to meet and solve people's various educational needs and social problems and provide some data reference and support for its future adult education and lifelong education.

## 2. Connotation of Community Education

### 2.1. Significance of Community Education from Marx's Perspective

Education in the process of human survival is a kind of cultivation process that has been implemented with growth since childhood. In this process, our personal thoughts and growth plans, as well as spiritual values, social values, and world values, are constantly maturing. From the growth of a single individual to drive the growth of the family and build social maturity and progress, the progress and development from a small family to everyone, to a country, and to the world are all from a single individual. Countries have been constantly exploring and studying the development and innovation of education. In the development of modern society, with the occurrence of aging social phenomena, social countries implement adult education and elderly reeducation models in education. From the traditional nine-year compulsory education to university education and even elderly education, many education models and methods have emerged. In this environment, the teaching mode of community education has been formed by following the main principles of Marx's thought, Lenin's thought, and Mao Zedong Thought and the form of socialist social development. With the progress of science and technology, the development of the Internet has not only driven more economic development and political value but also provided more help and guidance in the education mode and development path. According to Shengcong et al., community teaching has the characteristics of sociality, education, and politics. In the development and construction of cities, the development of community teaching mode is the inevitability of social development to a certain extent and the inevitability of people's pursuit of lifelong education [9]. Wei and Xujun developed this educational model, which is conducive in improving the overall quality of the people and establishing correct ideological values. People's thirst for knowledge can be realized and obtained from both horizontal and vertical under this educational platform. Using big data technology can better obtain the required knowledge content [10].

Figure 1 shows the community education platform. Community education not only has no requirements on the age and academic qualifications of students but also has diversified training types, such as entrepreneurship training, technical guidance, family education, and fire protection publicity, which play a lot of roles in improving the skills of students, and the improvement of community residents' skills promotes the development of the city.

### 2.2. Development and Curriculum Value of Community Education

In China, due to different regions, the economic level and environmental development of various regions are inconsistent, resulting in different maturity of community education, and the teaching results are also inconsistent. This teaching model has achieved good results in economically developed regions in China and has also developed well in provinces and cities in the central region; in the other remote mountainous rural areas, due to its remoteness, poor natural conditions, sparse population, low living standards, backward education, and the lack of support or maturity of policies, the development of education model is not ideal. This situation is most prominent in the western region of China, and its education development is relatively slow. Under the environment of big data and technical support, people's knowledge needs for various industries and fields are inconsistent, and the knowledge pursuit of adults and the elderly is also different. In terms of building community education subjects and resource reserves, through big data technology, we can more closely combine multiple disciplines and knowledge reserves to carry out differentiated education, and teachers can carry out online education and regular live teaching. It can effectively improve the initiative of educators. Macroscopically, the community teaching mode of adult education, on the one hand, plays a positive role in building personal national sense of honor and social responsibility and improving personal comprehensive quality; on the other hand, it provides more directions for the teaching methods of developing and innovating the national adult education mode from point to surface. Due to the wide range of choices in the curriculum, the temporal and spatial nature of the vertical learning direction is relatively free. It makes the learning time from adults to the elderly more free and has greater interest in learning. According to Zhong, with the rise of community education, while learning, it also plays a role in promoting the governance and management mode of the community. In life, common education can effectively promote the feelings of mutual help among residents. With the support of policies, it plays an important role in opening a happy garden and building ecological civilization in the future [11]. Chenxi put forward his imagination for the free and harmonious development and learning of people and knowledge, people and society, and people and the environment by opening the restrictions of inheritance and teaching to promote the new education mode of community education, aiming at developing the teaching mode with community characteristics to liberate the silent education environment, break the inherent educational concept wall, and create a community education ecosystem with humanistic care mode [12].

## 3. Community Education Curriculum Development under Big Data

### 3.1. Value of Community Education Courses under Big Data Technology

In the development and application of community education platforms, online teaching methods and resource search and processing are the main learning methods; the “online teaching” mode breaks the traditional teaching methods; allows us to directly obtain valuable resources on the Internet without considering the problems of downloading, saving, format conversion, and so on; simplifies the cumbersome steps of using network resources in real classes; and is the main way for us to accurately find educational resources and corresponding platform instructors that meet our personal needs in the vast data network platform. The complexity and diversity of user groups and the direction of knowledge needs are inconsistent. Diversified knowledge needs to be unified in a platform processor, which is a huge challenge to the ability of processors and digital computing. In this environment, big data technology is an inevitable need that can be handled as a whole. Under the condition of big data technology, the speed of data analysis and processing is faster. The planning classification of the management platform is more clear and specific. Because the huge data volume provides data support for further analysis and research, and there are many classifications of data, such as audio, video, pictures, text, PPT, geographical location, and other information. In the huge data processing, the required data can be accurately identified. On the education platform, the integration, analysis and processing of data, data analysis and mining, data sharing, and data presentation can be displayed in the form of visual reports, which makes people more intuitive about information screening and statistical analysis. In terms of system carrying capacity, it can also meet the needs of a large number of users online at the same time. Using the advanced technology of big data can provide more construction ideas for community education and provide more technical support for the development of the platform.

### 3.2. Research on the Path of Curriculum Development under the Big Data Environment

Based on the development of community courses in the big data environment and Marx's vision, there are serious deficiencies in platform management and information processing in the traditional network environment. Due to the inconsistent demand direction of community residents, the branch of information search is narrow. In the background processing, the system can only carry out data statistics based on the courses with a large audience, and the data analysis of minority clicks and selected courses is not accurate enough. There is no specific division and education for the universality and comprehensiveness of community education. In the big data processing technology, compared with the platform independent processing system in the traditional mode, the collection and aggregation ability of decentralized information in the platform management can be statistically processed and visual charts of data reports can be made. Managers can modify and improve the curriculum according to the collection and analysis of big data, meet the residents' diversified knowledge choice to the greatest extent, and provide higher technical support and means for the development path research in curriculum management. The establishment of an excellent education platform also makes the audience group of the platform more united and stronger, which is also beneficial to the unity of community residents, the authority of the platform, and the management mode of the platform. The establishment of friendly exchange and learning groups with friendly coexistence of residents plays a positive role in cultivating excellent talents and establishing a correct and positive sense of social responsibility and social values.

### 3.3. Research on the Development Path of Community Education Curriculum under Different Technologies

With the promotion of education and the popularization of the Internet, the trend of digital development of community education is becoming more and more obvious. For community education, big data also has unique characteristics. Community education takes community personnel as the object of education and provides them with learning opportunities. Based on the development of community education curriculum, the community education curriculum is comprehensively analyzed from four aspects according to the acceptance of community education under different technologies, and Table 1 is obtained.

In Table 1, through the acceptance of education courses under different technologies in the above table, it is obvious that the acceptance of using big data technology is stronger, and the overall data are higher than traditional technologies, making people learn efficiently with the help of big data.

In order to better compare the acceptance of community education courses under different technologies, we visualize the data in Table 1 to get Figure 2.

As shown in Figure 2, the visualization of the acceptance of community education courses under different technologies can clearly see the gap between big data technology and traditional technology, so as to more intuitively see the practicality of big data, improve the application ability of information technology, change the previous education mode, and realize the effective use of community education.

### 3.4. Research on the Development Path of Community Education Curriculum from Different Perspectives

With the continuous development of society, community training is also paid more and more attention. Therefore, an education system is gradually established to provide learning opportunities for the unemployed and those with low academic qualifications in the community, establish a resource platform for lifelong learning, and improve the education system with the educational platform goal of community construction. With the rapid development of the times, education is becoming more and more convenient. According to the analysis and research on the development path of community education courses from different perspectives, Table 2 is obtained.

In Table 2, through the research on the development path of educational curriculum under the different technologies in the above table, it is obvious that in Marx's vision, whether online or offline, teaching quality, knowledge reserve, or curriculum division, all the data are higher than that in the ordinary vision, which is enough to illustrate the influence of Marx's vision on it.

In order to better compare the path development of community education courses from different perspectives, the visualization is carried out according to the data in Table 2, and Figure 3 is obtained.

Figure 3 shows the development visualization of community education courses from different perspectives. The ups and downs of the data can clearly compare the impact on community education from Marx's perspective. Therefore, promoting community education from this perspective is the most important task for comprehensively improving the quality of the public.

### 3.5. Research on Curriculum Development of Community Education in Different Ways

Education is the top priority of our country and the foundation of our country. The education of a nation can reflect the state of the country. Therefore, as the country attaches importance to education, the mode of education is also changing. People of all ages are on the way of learning, and the learning method is not limited to schools and parks. Under the background of the development of education, a comprehensive analysis is made from the curriculum content, teaching mode, and teaching philosophy according to general adult education and community education, as shown Table 3.

Table 3 shows the data of curriculum development of curriculum education in different ways. In each performance, it can be seen that community education is significantly better than ordinary adult education. For education, it creates an education platform conducive to physical and mental health for teenagers and the elderly.

In order to better evaluate and compare the curriculum development of curriculum education in different ways, the visualization is carried out according to the data in Table 3, and Figure 4 is obtained.

Figure 4 shows the visualization of the performance evaluation of community curriculum education in different ways. It is very intuitive to see that community education courses are more popular; further enrich the amateur life of community teenagers, children, adult groups, and elderly groups; promote the community to carry out various colorful activities more actively; and play an application role in inheritance, civilization, value, etc.

## 4. Discussion

Through the research and analysis of the community education curriculum development from Marx's perspective under the big data environment, this paper can see that in the process of national development, education follows the lifelong teaching mode, which has a certain positive effect on people's ideological and political concepts and the direction of cultivating talents. Excluding the traditional education mode, the application of community education under big data technology improves the education development platform and data processing ability, so that the selection of courses and the reserve of knowledge are more suitable for the public, and the training of age, gender, and comprehensive quality has been improved and developed. In the development of education mode in the new era, there are still some deficiencies in the implementation policy of community education in China for the acceptance of the Internet to the application of science and technology in the development of various education fields and the opening of a new education environment. At present, the implementation effect in economically developed areas is relatively successful, and there are still deficiencies and technical deficiencies in the development of education in remote areas. The development direction of socialism in our country follows the advanced social concept of Marxism, and we should also keep pace with the times in the cultivation of people's educational thoughts and pursue the establishment of a knowledge exchange circle and learning circle for mass groups. Based on the online and offline development mode, community education can not only meet the needs of individuals but also provide more data reserves and statistics for community unity and social management. In this social platform, the education mode integrating learning, communication, making friends, and other functions breaks the traditional silent education mode for the freedom of education, so that knowledge can be liberated, people's minds can be liberated, and social development can also open up new development directions.

## 5. Summary

Community education curriculum is the key and important medium to promote the achievement of community education goals. Through research and exploration of this paper, in the existing social development, the development of digital economy and the application of big data technology have been combined, and certain breakthroughs and innovations have been made in the development of new educational models and curriculum development under the educational concept based on Marx's thought. People tend to live and use the Internet, which is in the rapid progress of the development of the Internet era. Through the network environment, the people of the country will be coordinated to build a learning ecosystem and a circle of friends, not only to effectively improve personal quality education and cultural level but also help individuals establish correct social outlook, values, and ideological quality. Based on the current direction of curriculum development, we should make use of the advantages of big data in the future development path to create a more flexible curriculum education and hierarchical education structure system that meet people's needs for adult education, provide more data support for the development of community education, and make a positive data basis for national policy support.

## Figures and Tables

**Figure 1:** Community education platform.

**Figure 2:** Visual diagram of acceptance of community education courses under different technologies.

**Figure 3:** Visual diagram of community curriculum education development from different perspectives.

**Figure 4:** Visual diagram of curriculum development of community curriculum education in different ways.

**Table 1:** Acceptance of community education courses under different technologies.

Acceptance level	Online and offline	Teaching quality	Knowledge reserve	Curriculum division
Traditional technology	40%	50%	45%	60%
Big data technology	60%	75%	70%	68%

**Table 2:** Research on the development path of community education curriculum from different perspectives.

Grouping	Ideological improvement	Educational evaluation	Spiritual ecology	Social values
From the traditional perspective	59	50	60	45
From the perspective of Marx	77	75	68	80

**Table 3:** Research on curriculum development of community education in different ways.

Grouping	Content of courses	Teaching model	Teaching philosophy
General adult education	55	48	58
Community education	60	59	70

## Data Availability

The data underlying the results presented in the study are available within the manuscript.
